# Deep Learning-Based Surface Nerve Electromyography Data of E-Health Electroacupuncture in Treatment of Peripheral Facial Paralysis

**DOI:** 10.1155/2022/8436741

**Published:** 2022-05-31

**Authors:** Pengdong Zhu, Hui Wang, Lumin Zhang, Xuan Jiang

**Affiliations:** ^1^Department of Acupuncture and Rehabilitation Physiotherapy, Ningbo Fenghua People's Hospital Medical Community, Ningbo, 315500 Zhejiang, China; ^2^Department of Electromyography, Ningbo Fenghua People's Hospital Medical Community, Ningbo, 315500 Zhejiang, China

## Abstract

This study was aimed at exploring the application value of electroacupuncture in the treatment of peripheral facial palsy using surface nerve electromyogram (EMG) image data based on deep learning. The surface nerve EMG recognition model was constructed based on multiview convolutional neural network, and the differences between it and the traditional single-view convolutional neural network were analyzed. Meanwhile, the influence of the multiview aggregation method based on pooling of view and decision fusion on facial recognition accuracy was compared and analyzed. 150 patients with peripheral facial paralysis were randomly divided into the control group (*n* = 70, basic treatment) and treatment group (*n* = 80, basic treatment + electroacupuncture). After 4 weeks of treatment, the therapeutic effect was evaluated by surface EMG parameters based on Horsfall-Barratt (*H*-*B*) scale and multiview convolutional neural network. The results showed that the face recognition accuracy of multiview convolutional neural networks was significantly higher than that of all single-view convolutional neural networks. The multiview aggregation network proposed in this research had a higher accuracy in facial recognition than the pooling of the view method and decision fusion-based multiview aggregation method. According to the evaluation results of H-B scale, the number of patients who recovered, significantly effective, effective, and ineffective in the control group was 39, 17, 3, and 11, respectively. The number of patients in the treatment group who recovered, significantly effective, effective, and ineffective was 51, 15, 9, and 5, respectively. Total effective rate of patients in the control group was 84.29%, and that of the treatment group was 93.75%, which was significantly higher than the control group (*P* < 0.05). According to surface EMG assessment results, compared with the control group, the mean root mean square (RMS), median frequency (MF), and mean power frequency (MPF) of the buccal and frontalis muscles in the treatment group increased significantly (*P* < 0.05). Compared with that before treatment, the mean buccal and frontalis RMS of patients in the control and treatment groups increased significantly after treatment (*P* < 0.05). In conclusion, electroacupuncture treatment could significantly improve the muscle strength of patients with peripheral facial paralysis.

## 1. Introduction

In recent years, deep learning, as a new machine learning method, has gradually attracted people's attention in the field of surface EMG based human-machine interface. Deep learning has the learning ability and can automatically learn features of different levels of abstraction from massive input samples. Thus, complex and tedious process of artificial signal feature extraction and optimization is avoided, and end-to-end EMG face recognition is realized [1]. Convolutional neural network is a deep neural network model widely used in the field of human-machine interface. The input data can be extracted layer by layer through multiple convolutional layers to extract abstract features. Through the pool layer between the convolution layers, features are downsampled, which greatly reduces the total training parameters and learns abstract features [2]. However, different types of convolutional neural networks have different effects in EMG face recognition.

E-health generally refers to the various applications of information and communication technology in medical treatment, including not only the informatization of medical procedures in hospitals but also the sharing of regional medical information and health services [3, 4]. E-health combined with traditional Chinese medicine is currently a research hotspot in the field of traditional Chinese medicine. Acupuncture is a commonly used treatment method in traditional Chinese medicine, which has a very good effect in the treatment of peripheral facial paralysis [5, 6], and is one of the dominant diseases in acupuncture treatment. The clinical manifestations of peripheral facial paralysis are incomplete eyelid closure and crooked mouth angles. It is mainly caused by inflammation of the facial nerve, commonly known as facial paralysis. The onset is often sudden, but most patients have a history of blowing, cold, or overwork before the onset. It is one of the clinical obstetric diseases, accounting for 60%-75% of all facial paralysis, and there are 450 cases per 100,000 people in China [7]. In recent years, the pathogenesis of peripheral facial paralysis, the pathological changes after the onset, and the principles of clinical treatment have been the main difficulties for medical researchers and clinicians to overcome. At present, the treatments of western medicine are mainly rehabilitation, oral medication, and surgery, while the curative effect of acupuncture and moxibustion of traditional Chinese medicine on peripheral facial paralysis has been confirmed [8]. However, there are often different controversies in the evaluation of its efficacy. Surface EMG adopts surface electrodes to be placed on the patient's target muscle to understand the overall effect of neuromuscular activity. Compared with traditional needle EMG, it has larger detection space and good repeatability and thus widely used in the evaluation of facial nerve and muscle function [9, 10]. However, there is very little research on the clinical application of peripheral facial paralysis evaluation.

Therefore, the adoption of surface nerve EMG recognition data analysis based on multiview convolutional neural network in the treatment of peripheral facial paralysis by E-health electroacupuncture and its clinical effect was explored, to provide a scientific basis for the clinical adoption of surface EMG in facial paralysis.

## 2. Materials and Methods

### 2.1. Surface Nerve EMG Recognition Based on Multiview Convolutional Neural Network

The multiview convolutional neural network is mainly composed of two parts. The first part is a multistream convolutional neural network composed of multiple branches. Each branch is modeled separately for each view data, in which it can make full use of each view information in the learning process. The second part adopts the multiview aggregation network to aggregate the multiview features learned in the first part of the network.

Part I is as follows: multistream convolutional neural network structure. Each branch of the multistream convolutional neural network mainly contains two convolutional layers: two locally connected layers and one fully connected layer.  Table 1 is the hyperparameter setting of the multistream convolutional neural network. The ReLU nonlinear activation function and batch normalization are adopted for each layer of the multistream convolutional neural network, and Dropout is adopted after the fourth layer of the network.

Part II is as follows: the structure of multiview aggregation network. The multiview aggregation network consists of two subnetworks: the preaggregation and postaggregation network. In Figure 1, in the preaggregation network, the multiview features output by the first convolutional layer of the three branches of the multistream convolutional neural network will be fused by the feature layer. The input will be processed by one convolutional layer, two locally connected layers, three fully connected layers, and a softmax classification function to form an aggregation network for multiview aggregation. In the postaggregation network, the multiview features output by the first fully connected layer of the three branches of the multistream convolutional neural network will be fused by the feature layer. The input will be processed by two fully connected layers and one softmax classification functions to form an aggregation network for multiview aggregation. The hyperparameter settings of the preaggregation network and the postaggregation network are shown in Tables 2 and 3. ReLU nonlinear activation function and batch normalization are adopted for each layer of the two subnetworks. Meanwhile, Dropout is adopted at the third and fourth layers of the preaggregated network.

It is assumed that the output feature of the *i*-th convolutional neural network and the *j*-th hidden layer is *H*_*i*_^*j*^, and then preaggregation network and postaggregation network can be written as the following equations (1) and (2), respectively.

(1) $$\begin{array}{c} H_{\text{input}-\text{pre}-\text{fusion}}=\theta \left(f{\text{use}}_{F}\left(H_{i}^{1}，i=1,2,3\right)\right), \end{array}$$

(2) $$\begin{array}{c} H_{\text{input}-\text{post}-\text{fusion}}=\theta \left(f{\text{use}}_{F}\left(H_{i}^{5}，i=1,2,3\right)\right). \end{array}$$

*f*use_*F*_ represents the fusion operation of the feature layer, and *θ*( ) represents the nonlinear activation function of ReLU.

The face image category probability vectors output by the preaggregation network and the postaggregation network are *y*_pre−fusion_ and *y*_post−fusion_, which are then merged through the decision layer, and the final facial recognition result *y*_final_ is as follows.

(3) $$\begin{array}{c} y_{\text{final}}=y_{\text{pre}-\text{fusion}}+y_{\text{post}-\text{fusion}}. \end{array}$$

The performance of multiview convolutional neural network and single-view convolutional neural network is compared and analyzed. The structure of single-view convolutional neural network is shown in Figure 2 below.

### 2.2. Construction of Different Multiview Aggregations

By comparing pooling of view-based multiview aggregation and decision fusion-based multiview aggregation, the impact of different multiview aggregations on the accuracy of facial recognition is analyzed. The structure diagram of multiview aggregation based on pooling of view is shown in Figure 3 below. This view aggregation method is close in principle to the pooling layer in convolutional neural network; so, it is called pooling of view. The structure diagram of multiview aggregation based on decision fusion is shown in Figure 4. This view aggregation method mainly constructs a softmax classification function for network branches that process different view data. Then, the classification result is obtained in the form of the probability vector of the facial image category. Finally, the facial image category probability vectors are output to multiple branches, and the decision-making layer fusion is performed, after which the facial image classification result is obtained.

### 2.3. General Clinical Information

150 patients with peripheral facial nerve palsy admitted to hospital from May in 2014 to May in 2019 were selected. They were in line with the diagnostic criteria of *Traditional Chinese Medicine Internal Disease Diagnosis and Treatment Routines* and Western medicine's *Internal Disease Diagnostic Standards*. All patients were randomly divided into the control group and treatment group. In the control group, there were 70 cases, 37 males, and 33 females. The age range was (21-55) years, and the course of disease was (7-15) days. There were 80 cases in the treatment group, including 42 males and 38 females. The age range was (20-53) years, and the course of disease was (7-14) days. There was no significant difference between the two groups of patients in general information such as age, gender, and disease course. This study was approved by the ethics committee of hospital, and all the enrolled patients were informed and consented.

Inclusion criteria were as follows: (I) patients meeting the diagnostic criteria of Traditional Chinese and Western medicine; (II) patients aged between 8 and 60 years old; and (III) patients voluntarily participated in the study after being informed.

Exclusion criteria were as follows: (I) the patient was in pregnancy or lactation; (II) the patient had previous cardiovascular and cerebrovascular diseases, liver and kidney insufficiency, or hematopoietic dysfunction; (III) patients with facial palsy, Guillain-Barre syndrome, ear disease, Ramsay Hunt syndrome, and other diseases caused by central nervous system; and (IV) patients who cannot accept or adhere to the treatment in this study.

### 2.4. Treatments

Both groups of patients were treated with basic treatments of oral hormone shock therapy and nutritional nerve therapy.

The control group was as follows: patients were treated with basic treatment.

The treatment group was as follows: patients were treated with electroacupuncture and basic treatment. The patient was fixed in the supine position, with main acupoint temple, Yangbai, Quanliao, Dicang, chia ch'e, Xiaguan, and Sibai selected on the affected side, and needles were inserted by oblique thrusting. Fengchi acupoint was selected in both sides, and needles were inserted by neutral supplementation and draining method. Yifeng and Hegu were selected in both sides, and needles were inserted by the draining method. The needle was kept for 30 minutes and injected once every 5 minutes. The needles were “Hanyi Brand” acupuncture needles with a specification of 0.3 × 40 mm. The treatment device was the Hwato SDZ-II electronic acupuncture treatment device.

Two groups of patients were treated for 4 weeks, and then the treatment effect was evaluated. During the treatment, the two groups of patients did not use other drugs, so as not to interfere with the treatment effect.

### 2.5. Observation Indexes

(I) *H*-*B* scale was as follows: the *H*-*B* facial nerve function evaluation system recommended by the International Neurosurgery was adopted to evaluate the facial nerve function. There were four types of scoring: recovery, significantly effective, effective, and ineffective, and the specific scoring content was in Cao's literature [11]. (II) Surface EMG was as follows: FlexComp Infiniti type surface EMG analyzer was used, and its surface nerve EMG recognition function was optimized by multiview convolutional neural network. The optimized surface EMG analyzer was adopted to collect surface EMG signals of the frontalis and buccinator of patients before and after treatment. The signal processing software of the surface electromechanical equipment was adopted for analysis and processing. Indicators included RMS that reflected muscle strength, MF that referred to the median value of the frequency of electrical discharge along muscle fibers during skeletal muscle contraction, and MPF that reflected the conduction speed of peripheral motor potentials and the types of motor units participating in activities and the degree of synchronization.

### 2.6. Statistical Analysis

MATLAB (2017 version) software was adopted to analyze EMG signal in time domain and frequency domain. All measurement data were expressed as mean plus or minus standard deviation, and count data were expressed as the number of cases (percentage). Statistical analysis was performed by SPSS software. The comparison of measurement data between the two groups was performed via *t*-test, and the comparison of count data between the two groups was performed via chi-square test. *P* < 0.05 meant the difference was statistically significant.

## 3. Results

### 3.1. Performance Comparison between Multiview and Single-View Convolutional Neural Network

In Figure 5, the accuracy of the multiview convolutional neural network in facial recognition was significantly higher than that of all single-view convolutional neural networks, which indicated that the multiview convolutional neural network had higher performance in facial EMG image recognition than the traditional single-view convolutional neural network. In addition, in terms of accuracy of face recognition, the single-view convolutional neural network (column 2) splicing multiview data was 87.3, and the difference between single-view convolutional neural network (column 3 87.1, column 4 87, column 5 87.1) and single-view convolutional neural network of single-view data was very small, which showed that in the recognition of facial EMG image, the single-view convolutional neural network method that splices multiple view data could not effectively improve the performance.

### 3.2. Performance Comparison of Different Multiview Aggregations

From Figure 6, the proposed multiview aggregation network could obtain higher accuracy in facial recognition than pooling of view-based multiview aggregation and decision fusion-based multiview aggregation. In addition, after the second FC, the facial recognition accuracy of multiview aggregation based on pooling of view and the multiview aggregation network proposed in this research was close (88% vs 88.2%), and the difference was only 0.2%. It meant that the multiview aggregation based on pooling of view after the second FC also had higher performance in facial EMG image recognition.

Red: the multiview aggregation network proposed in this research, blue: multiview aggregation based on pooling of view, and green: multiview aggregation based on decision fusion.

### 3.3. Evaluation of *H*-*B* Facial Nerve Function after Treatment in the Two Groups

In Figure 7, the number of patients in the control group who were recovered, significantly effective, effective, and ineffective was 39, 17, 3, and 11, respectively. The number of patients in the treatment group who were recovered, significantly effective, effective, and ineffective was 51, 15, 9, and 5, respectively. The statistical results of the total effective rate of the two groups of patients were shown in Figure 8. Compared with the control group, the total effective rate of patients in the treatment group increased significantly (*P* < 0.05), and the difference was statistically significant.

### 3.4. Comparison of Surface EMG Parameters before and after Treatment between the Two Groups

The comparison of the mean RMS of surface EMG parameters before and after treatment between the two groups of patients was shown in Figure 9. Compared with the control group, the mean values of RMS of buccinator and frontalis in the treatment group increased significantly (*P* < 0.05). Compared with that before treatment, the mean RMS of buccinator and frontalis of patients in the control and treatment groups increased significantly after treatment (*P* < 0.05).

The comparison of the maximum value of the surface EMG parameter RMS between the two groups of patients before and after treatment was shown in Figure 10, and there was no significant difference in the maximum value of RMS of buccinator and frontalis between the two groups of patients before and after treatment.

The comparison results of surface EMG parameters MF before and after treatment between the two groups of patients were shown in Figure 11. Compared with the control group, the MF of buccinator and frontalis of the treatment group increased significantly (*P* < 0.05). Compared with that before treatment, the MF of buccinator and frontalis of the control group and the treatment group increased significantly after treatment (*P* < 0.05).

The comparison results of the surface EMG parameters of MPF of patients before and after treatment were shown in Figure 12. Compared with the control group, the MPF of buccinator and frontalis of the treatment group were significantly increased (*P* < 0.05). Compared with that before treatment, the MPF of buccinator in the control group increased significantly after treatment (*P* < 0.05), and the MPF of buccinator and frontalis in the treatment group increased significantly after treatment (*P* < 0.05).

## 4. Discussion

The surface EMG signal is a kind of bioelectric signal, which is collected by electrodes placed on the surface of the skin. Its essence is that human muscle contraction is the superposition of action potentials of all motor units in the area where the electrode covers the muscle. It can reflect the activity state of human muscles and nerves [12]. Facial recognition based on surface EMG requires machine learning methods to train a classifier model for facial image classification and recognition. The traditional machine learning facial EMG image recognition method mainly relies on manual extraction of EMG signal features, and the quality of the selected features often directly affects the final facial recognition performance [13]. To improve the performance of facial EMG image recognition, a multiview deep learning method was proposed. The multiview data of the EMG signal was constructed by extracting the EMG signal feature set, which was proved to be better than the traditional single view in performance. It indicated that the multiview convolutional neural network had higher performance in facial EMG image recognition than the traditional single-view convolutional neural network. In addition, the single-view convolutional neural network method that splices multiple view data could not effectively improve the facial recognition performance. According to the performance comparison study of different multiview aggregations, it was found that the proposed multiview aggregation network could obtain higher accuracy in facial recognition than pooling of view-based multiview aggregation and decision fusion-based multiview aggregation. This was consistent with previous studies [14, 15], indicating that surface nerve EMG recognition based on multiview convolutional neural network had higher performance. Thus, it was better than pooling of view-based multiview aggregation and decision fusion-based multiview aggregation and had obvious advantages in clinic.

At present, there is no uniform standard for the evaluation scale of peripheral facial paralysis. The *H*-*B* scale is the most widely adopted in acupuncture clinical research. Research reported that surface EMG for evaluating peripheral facial paralysis was highly correlated with the *H*-*B* scale [16, 17], indicating that surface EMG could be taken to evaluate the efficacy of peripheral facial paralysis. The number of patients who recovered, significantly effective, effective, and ineffective in the control group was 39, 17, 3, and 11, respectively. The number of patients in the treatment group who recovered, significantly effective, effective, and ineffective was 51, 15, 9, and 5, respectively. Compared with the control group, the total response rate in the treatment group was significantly higher (*P* < 0.05), and the difference was statistically significant. This was consistent with previous research results [18], which meant that electroacupuncture had a significant effect in the treatment of peripheral facial paralysis. Moreover, the role of *H*-*B* scale in the evaluation of the efficacy of peripheral facial paralysis was confirmed. The evaluation effect of the efficacy of surface EMG on peripheral facial paralysis was compared and analyzed, and the mean RMS of buccinator and frontalis of patients in the treatment group increased significantly compared with those of the control group. Compared with that before treatment, the mean RMS of buccinator and frontalis of patients in the control group and the treatment group increased significantly after treatment. There was no significant difference in the maximum RMS of buccinator and frontalis between the two groups of patients before and after treatment, which was consistent with the previous results [19].

RMS reflects the level of muscle discharge within a certain period of time, which is believed to be related to the number of motor units recruited and the synchronization of muscle fiber discharge, and is often used to detect muscle activity time and assess muscle strength [20]. The results showed that after treatment, the average RMS of buccal muscle and front of rontal muscle was 18.42 ± 2.4 *μ*V and 10.51 ± 2.2 *μ*V in the control group and 24.67 ± 2.4 *μ*V and 16.42 ± 2.2 *μ*V in the treatment group, respectively. The mean RMS in the treatment group increased significantly (*P* < 0.05). In addition, the mean RMS in both groups increased significantly after treatment compared with before treatment (*P* < 0.05). After electroacupuncture, the patient's muscle activation increased, and muscle contraction improved, but the maximum value of RMS did not change significantly. It showed that there was no change in the maximum muscle contraction force, which was a point to be concerned about in subsequent studies. After treatment, the buccinator and frontalis MF values were 89.5 ± 10.8 Hz and 94.2 ± 10.4 Hz in the control group and 108.4 ± 10.6 Hz and 115.4 ± 10.4 Hz in the treatment group, respectively, which significantly increased (*P* < 0.05). The MPF values of buccinator and frontalis in the control group were 112.4 ± 8.6 Hz and 104.3 ± 7.9 Hz, respectively, and those in the treatment group were 143.5 ± 8.2 Hz and 125.9 ± 7.8 Hz, respectively (*P* < 0.05). MPF was related to the activity of muscle fiber units, and its increase indicated that paralyzed muscles started to move, indicating that peripheral facial paralysis was improved [21].

## 5. Conclusion

Surface nerve EMG recognition based on multiview convolutional neural network was of high performance in evaluating the efficacy of electroacupuncture-treated peripheral facial paralysis, which was better than traditional single-view convolutional neural network. After 1 month of electroacupuncture, there were significant therapeutic effects in peripheral facial paralysis patients, and the muscle strength of buccinator and frontalis had improved. However, there are still some limitations in this research, such as the small sample size and the fact that the therapeutic effect is not evaluated according to the age and condition of patients. However, this research can still provide scientific basis for the clinical adoption of surface EMG in facial paralysis.

## Figures and Tables

**Figure 1:** Schematic diagram of the multiview convolutional neural network structure. Conv: convolutional layer; LC: locally connected layer; FC: fully connected layer. The numbers after them represent the number of hidden units or convolution kernels, and the number after @ represents the size of convolution kernel.

**Figure 2:** Schematic diagram of single-view convolutional neural network structure.

**Figure 3:** Multiview aggregation based on pooling of view.

**Figure 4:** Multiview aggregation based on decision fusion.

**Figure 5:** Performance comparison between multiview and single-view convolutional neural network. Red: multiview convolutional neural network. Blue: single-view convolutional neural network.

**Figure 6:** Performance comparison of different multiview aggregations. Conv: convolutional layer, LC: locally-connected layer, FC: fully connected layer.

**Figure 7:** *H*-*B* scale scores of the two groups of patients after treatment.

**Figure 8:** Comparison of total effective rate via *H*-*B* scale scores between two groups of patients after treatment. ^∗^Compared with the control group, *P* < 0.05.

**Figure 9:** Comparison of the RMS mean values of the two groups of patients before and after treatment. ^∗^Compared with the control group, *P* < 0.05; # compared with that before treatment, *P* < 0.05.

**Figure 10:** Comparison of the maximum RMS between the two groups of patients before and after treatment.

**Figure 11:** Comparison of MF before and after treatment between the two groups. ^∗^Compared with the control group, *P* < 0.05; #compared with that before treatment, *P* < 0.05.

**Figure 12:** Comparison of MPF before and after treatment between the two groups. ^∗^Compared with the control group, *P* < 0.05; # compared with that before treatment, *P* < 0.05.

**Table 1:** Hyperparameter settings of multistream convolutional neural network.

Name of the view	Corresponding feature set	Recognition accuracy (%)	Name of the view	Corresponding feature set	Recognition accuracy (%)
View 1	Du feature set	82.6	View 6	Doswald feature set	85.4
View 2	Correlation of time domain operator	81.1	View 7	Discrete wavelet transforming coefficients	85.6
View 3	Atzori feature set	83.5	View 8	Discrete wavelet packet transforming coefficients	85.8
View 4	Phinyomark feature set 1	85.6	View 9	Continuous wavelet transforming coefficient	84.3
View 5	Phinyomark feature set 2	84.4	View 10	Hudgins feature set	82.6

**Table 2:** Hyperparameter settings of the preaggregation network.

Hidden layer		Hyperparameter		Hidden layer		Hyperparameter	
Name	Type	Name	Setting	Name	Type	Name	Setting
First layer	Convolutional layer	Size of convolution kernel	3 × 3	Third layer	Local connection layer	Number of convolution kernels	64
First layer	Convolutional layer	Number of convolution kernels	64	Fourth layer	Fully connected layer	Number of hidden units	512
Second layer	Local connection layer	Size of convolution kernel	1 × 1	Fifth layer	Fully connected layer	Number of hidden units	512
Second layer	Local connection layer	Number of convolution kernels	64	Sixth layer	G-way fully connected layer	Number of hidden units	Number of facial images to be classified
Third layer	Local connection layer	Size of convolution kernel	1 × 1	Seventh layer	Softmax classification function	—	—

**Table 3:** Hyperparameter settings of the postaggregation network.

Hidden layer		Hyperparameter	
Name	Type	Name	Setting
First layer	Fully connected layer	Number of hidden units	512
Second layer	G-way fully connected layer	Number of hidden units	Number of facial images to be classified
Third layer	Softmax classification function	—	—

## Data Availability

The data used to support the findings of this study are available from the corresponding author upon request.
